The article "Radiomics Analysis on Noncontrast CT for Distinguishing Hepatic Hemangioma (HH) and Hepatocellular Carcinoma (HCC)" was published in 2022. Journal: Contrast Media Mol Imaging.

# Radiomics Analysis on Noncontrast CT for Distinguishing Hepatic Hemangioma (HH) and Hepatocellular Carcinoma (HCC)

**DOI:** 10.1155/2022/7693631

**Published:** 2022-06-25

**Authors:** Shuyi Hu, Xiajie Lyu, Weifeng Li, Xiaohan Cui, Qiaoyu Liu, Xiaoliang Xu, Jincheng Wang, Lin Chen, Xudong Zhang, Yin Yin

**Affiliations:** ^1^Department of Hepatobiliary Surgery, Nanjing Drum Tower Hospital Clinical College of Nanjing Medical University, Nanjing, China; ^2^First Clinical Medical College of Nanjing Medical University, Nanjing 210029, China; ^3^Weifang Medical University, Weifang 261053, China; ^4^School of Electronic Science and Engineering, Nanjing University, Nanjing 210046, China; ^5^Department of Hepatobiliary Surgery, Nanjing Drum Tower Hospital, The Affiliated Hospital of Nanjing University Medical School, 321 Zhongshan Road, Nanjing 210008, Jiangsu Province, China; ^6^Department of General Surgery, Jiangsu Cancer Hospital & Jiangsu Institute of Cancer Research & The Affiliated Cancer Hospital of Nanjing Medical University, Nanjing 210009, China; ^7^Department of Hepato-biliary-pancreatic Surgery, The Affiliated Changzhou No. 2 People's Hospital of Nanjing Medical University, Changzhou, Jiangsu, China

## Abstract

**Background:**

To form a radiomic model on the basis of noncontrast computed tomography (CT) to distinguish hepatic hemangioma (HH) and hepatocellular carcinoma (HCC).

**Methods:**

In this retrospective study, a total of 110 patients were reviewed, including 72 HCC and 38 HH. We accomplished feature selection with the least absolute shrinkage and operator (LASSO) and built a radiomics signature. Another improved model (radiomics index) was established using forward conditional multivariate logistic regression. Both models were tested in an internal validation group (38 HCC and 21 HH).

**Results:**

The radiomic signature we built including 5 radiomic features demonstrated significant differences between the hepatic HH and HCC groups (*P* < 0.05). The improved model demonstrated a higher net benefit based on only 2 radiomic features. In the validation group, radiomics signature and radiomics index achieved great diagnostic performance with AUC values of 0.716 (95% confidence interval (CI): 0.581, 0.850) and 0.870 (95% CI: 0.782, 0.957), respectively.

**Conclusions:**

Our developed radiomics-based model can successfully distinguish HH and HCC patients, which can help clinical decision-making with lower cost.

## 1. Introduction

Hepatocellular carcinoma (HCC) is the second greatest threat that leads to cancer deaths all over the world, accounting for approximately 70% of primary liver cancers [1]. The incidence of HCC in the United States has almost tripled over the past 40 years [2, 3]. Even with appropriate treatments such as ablation and surgical resection, 50–60% of HCC patients still undergo tumor recurrence within a five-year period [4, 5]. Hepatic hemangioma is a regenerative neoplasm that rarely grows in volume, with a relatively lower risk of complications and favorable outcomes. Hematomas in small and medium sizes (0–3 cm, 3 cm–10 cm) usually do not require treatment [6, 7]. Therefore, classification via noninvasive methods between hepatic hemangioma (HH) and hepatocellular carcinoma (HCC) should be discovered and applied.

The differential diagnosis of HH and HCC is mainly based on serological tests, tumor markers, and imaging studies involving liver ultrasound (US), computed tomography (CT), and magnetic resonance imaging (MRI). Clinically, a contrast-enhanced CT scan is typically applied to distinguish HH from HCC. For instance, HH appears on scans as one or more clear nodules with low density on CT. After injecting contrast agents, an enhancement is present in nodule peripheral and homogeneous centripetal filling [8]. A rapid enhancement of hepatic artery and transient washout show a relatively high specificity with the diagnosis of HCC [9]. However, previous studies showed low sensitivity (almost 50%) especially for the lesion's diameter smaller than 1 cm [10]. Moreover, alpha fetoprotein (AFP), the most remarkable diagnostic serological marker, could also be at high levels in acute hepatitis, cirrhosis, colitis, etc. These lead to the challenges of the precise diagnosis of small-size HH or HCC [9, 11].

Radiomics, a new algorithm designed to extract and analyze image features, has experienced rapid development in cancer diagnosis in recent years [12]. Image analysis tools of radiomics come to aid in the precise and personalized diagnosis and treatment [13]. A retrospective study in 2019 that established a radiomics-based model to predict biliary tract cancers was found impressive in this field [14]. Despite its powerful instructive functions, how to improve the interpretability of radiomic features requires further research before a pervasive standard is set to distinguish HH from HCC patients [15]. The aim of this study is to build radiomics-based methods on noncontrast CT scans for distinguishing between HH and HCC.

## 2. Methods

This retrospective study was approved by the institutional review board of our hospital and the requirement for written informed consent was waived. All methods involved were performed in terms of relevant guidelines and regulations.

### 2.1. Patients

We searched our institution's medical records and obtained 291 cases of hepatic lesions preliminarily between January 1, 2016, and October 1, 2020. The exclusion criteria were as follows: (1) lack of exact HH or HCC pathological evidence (*n* = 20); (2) lack of standard abdominal noncontrast CT images (*n* = 17); (3) time spans between CT scans and the operation over three months (*n* = 33); and (4) lack of complete clinical information (*n* = 52). A total of 169 patients including HCC (110/169) and HH (59/169) were finally included in this study (Figure 1).

These patients all had clear pathological diagnoses after hepatectomy with postoperative care. We randomly (2 : 1 ratio) set up a training group by selecting 110 patients (72 HCC and 38 HH), and the remaining 59 patients (38 HCC and 21 HH) were in the validation group. All patients underwent noncontrast CT scans before the therapeutic schedules.

Relevant information was obtained from the patients' medical records. Clinical characteristics included age, sex, size of the lesion, number of lumps, and histological grade.

### 2.2. Pathological Analysis and CT Acquisition

Liver samples were analyzed by two pathologists with diverse clinical experience (2.5 and 5 years, respectively). Both of them were blinded to the medical details of the study cohort.

The workflow is displayed in Figure 2. All CT examinations were performed on the same model CT scanner (Lightspeed, VCT, or Discovery HD 750, GE Health Care, US). The parameters were unified (tube voltage 120 kVp, tube current 250–350 mA, collimating slice thickness of 5 mm, reconstruction slice thickness of 1.25 mm, slice interval 5 mm, rotation time 0.6 s, helical pitch 1.375, the field of view between 35 and 40 cm, and matrix 512 × 512) and the same reconstruction algorithm was applied.

### 2.3. Image Segmentation and Radiomic Features Extraction

Two radiologists reviewed the noncontrast CT images of all patients and extracted radiomic features. They evaluated the shape and size of lesions and drew along the tumor contour (region of interest (ROI)) on each layer (volume of interest (VOI)) with the 3D slicer software (version 4.10.2; https://www.slicer.org). The preprocessing and image feature extraction were performed using the Pyradiomics package (https://www.radiomics.io/pyradiomics.html). Eight hundred forty radiomics features including 18 first-order statistics, 74 textural ones, and 758 wavelet-based transformations, were calculated based on every VOI. Z-scores were applied to normalize the values of features in both the training and validation groups. To measure each feature's reproducibility, intraobserver and interobserver intraclass correlation coefficient (ICC) were applied in this process, adopting 50 randomly picked cases. To assess intraobserver reliability, Reader 1 accomplished image segmentation independently and Reader 2 repeated the similar process twice a week.

The selection of significant radiomic features was performed in the following steps. Features with high stability (intraobserver and interobserver ICC > 0.8) were kept. Next, the least absolute shrinkage and operator (LASSO) logistic regression was conducted with 10-fold cross-validation. A radiomics signature was formed as a linear composition of independent features due to respective coefficients.

### 2.4. Establishment of the Radiomics-Based Model

The forward conditional multivariate logistic regression was also involved. This reduces coefficients through penalizing correlated features to cope with multicollinearity problems. Independent features were selected to constitute the more precise radiomic index model.

### 2.5. Statistical Analysis

Categorical and continuous variables were compared with the *χ*2 test and Student's *t*-test, respectively. R software (version 3.6.2, https://www.r-project.org) was used for statistical analysis. The ROC curve and the area under the curve (AUC) value were applied to evaluate the performance of two different radiomics models (the radiomics signature and radiomics index). The calibration curves were computed via bootstrapping with 1000 resamples to evaluate the deviation between the predicted and actual value, accompanied by the Hosmer–Lemeshow test. The decision curve analysis (DCA) was applied in evaluating the net benefits provided by the radiomics-based models. *P* < 0.05 was indicative of statistical significance.

## 3. Results

### 3.1. Baseline Information

According to Table 1, no statistical differences were shown in patients between the training and validation groups. The training group included a total of 110 patients (72 HCC and 38 HH), and the validation group included 59 patients (38 HCC and 21 HH).

### 3.2. Performance of the Radiomics Signature

Five radiomic features (original-shape-volume, wavelet-LLL-first-order-median, wavelet-LLL-gldm-small-dependence-low-gray-level-emphasis, wavelet-LHL-glszm-zone-entropy, and wavelet-LLH-glszm-zone-entropy) with nonzero coefficients were chosen (Figure 3). Our radiomics signature was constituted with a formula based on selected radiomic features. The radiomics signature demonstrated performance with AUC values of 0.792 (95% confidence interval (CI): 0.703, 0.882) in the training group and 0.716 (95% CI: 0.581, 0.850) in the validation group (Table 2).

### 3.3. Establishment and Performance of the Radiomics Index

To elevate the predictive accuracy, we eliminated three features through the forward conditional multivariate logistic regression (Table 3). Only two features were further used to construct the radiomics index in the following formula. Radiomics index = 1.218 + 0.687 *∗* wavelet-LLL-first-order-median-2.165 *∗* wavelet-LHL-glszm-zone-entropy, in which first order represents the histogram of voxel intensity values, *and glszm (gray level size zone)* describes the linked voxels with identical gray-level intensity. Lower glszm zone entropy and higher median values of voxel intensity values might indicate more uniform pixels in the region of interest.

Boxplots of two models are shown in Figures 4(a) and 4(b). The radiomics index demonstrated greater performance with higher AUCs of 0.880 (95% CI: 0.817, 0.943) and 0.870 (95% CI: 0.782, 0.957) in the training and validation groups. The radiomics index achieved a sensitivity of 80.6% and 60.5%, with a specificity of 81.6% and 100%, a positive predictive value of 89.2% and 100%, and a negative predictive value of 68.9% and 58.3% in two groups, respectively (Table 2).

The calibration curve of models revealed consistency between the prediction and pathological outcomes, especially in the radiomics index (Figures 4(c) and4(d)). The DCA for the radiomics signature and radiomics index is shown in Figure 5. According to this figure, the radiomics index provided more clinical benefit for distinguishing HH and HCC than the radiomic signatures across the majority of the range of threshold probabilities in the validation cohort.

## 4. Discussion

With the increasing applications of radiomics, we aimed to develop radiomic-based models to assist clinical differentiation of HH and HCC. This study built up a radiological model to distinguish HH and HCC based on noncontrast CT-extracted features. The radiomics index included 2 main radiomic features, which were screened out through several steps and showed great performance to differentiate HH and HCC.

Pathologically, HCC evolves from dysplastic lesions (dysplastic foci/dysplastic nodules) with bleeding, calcification, and necrosis tissue [16, 17]. In contrast, HH stems from vascular malformation and contains rich sinusoids [18]. In noncontrast CT images, both the HCC and HH show similar low-density mass. The use of spectral CT can increase the sensitivity for differentiating small HHs from HCCs in the late arterial phase and portal venous phase [19, 20]. The status of clear boundaries distinguished HH from HCC. However, in clinical practice, the small lesions are indistinguishable according to macroscopic image findings. Previous studies investigated radiomics-based differentiation of HH and HCC through MRI-extracted features [21–23]. Moreover, these MRI studies applied machine learning techniques to the development of prediction models that made the model structure hard to understand. Although MRI and contrast CT images could offer more information, noncontrast CT images are more commonly performed in clinics. This study provided the first evidence for the discrimination ability of noncontrast CT features, and we used a simple formula that can be easily validated.

The reproducibility of radiomics features remained a worried issue due to the adverse effects of radiation dosage and CT reconstruction [24]. In order to solve this issue, we set up a reproducibility examination. Only 88 reproducibility features (intraobserver and interobserver ICC >  0.8) met the criteria among 840 radiomic features (18 first-order statistics, 74 textural ones, and 758 wavelet-based transformations). This might be explained by the different VOIs (ROI selection and growth or shrinkage of margin) sketched by two radiologists [25].

Jacob Sosna et al. suggested that fewer reproducible radiomic features illustrated better reproducibility [26]. These two radiomic features selected with the forward conditional multivariate logistic regression are wavelet-LLL-first-order-median and wavelet-LHL-glszm-zone-entropy. Both of them indicate uniform pixels of the gray level zones. These results might be highly consistent with the pathological differences between HH and HCC, in which HH consists of vascular malformation and HCC contains mainly cytological atypia.

Several limitations should be noted in this study. First, all the study information came from one single medical center and validation in multiple centers is necessary in further research. Second, due to the retrospective nature of our study, selection bias could not be avoided. Third, the limitations of clinical significance exist only in noncontrast CT scans. The application of ultrasound and other radiological images is worthy to be studied in the future.

In conclusion, we developed radiomics models to distinguish HH and HCC on the basis of radiomic features derived from noncontrast CT images. These radiomics-based models have the potential to assist clinical diagnosis and offer more radiological information with a noninvasive method.

## Figures and Tables

**Figure 1:** Patient selection flowchart.

**Figure 2:** Main working procedures in this research. (a) Volume of interest was individually depicted on CT images at each transverse. (b) Radiomic features include first-order statistics, textural ones, and wavelet transformations. (c) Intraobserver and interobserver reproducibility analysis and LASSO regression were applied in feature selection. (d) Radiomics-based models were established on the basis of selected features. (e) Calibration curves and decision curve analysis were used to evaluate diagnostic performance of two models.

**Figure 3:** Statistical selection process of radiomic features with LASSO regression. (a) Optimal *λ* value was calculated by LASSO model with 10-fold cross-validation. The binomial deviance curves were drawn versus log (*λ*). (b) Respective coefficient details were depicted. (c) Five features related to the optimal value were further reserved with respective coefficients to build the radiomics signature model.

**Figure 4:** Two models-radiomics signature and radiomics index were established using selected features. Comparisons of boxplots between the HH and HCC in radiomics signature (a) and radiomics index (b). Calibration curves of radiomics signature (c) and radiomics index (d).

**Figure 5:** Decision curve analysis of radiomics signature and radiomics index. The *Y*-axis represents the net benefit. The radiomics index provided more clinical benefits than treating all or none of the patients, and the radiomics signature.

**Table 1:** Baseline characteristics.

Parameter	Training (*n* = 110)	Validation (*n* = 59)	*P* value
Sex			0.32
No. of men	72 (65.5)	34 (57.6)	
No. of women	38 (34.5)	25 (42.4)	
Age (years)			0.15
<60	47 (42.7)	32 (54.2)	
≥60	63 (57.3)	27 (45.8)	
Laboratory findings			
ALT (IU/mL)	29.8 (23.0–42.3)	27.1 (22.1–37.8)	0.37
Total bilirubin (ng/mL)	12.4 (8.2–16.4)	12.3 (9.2–15.5)	0.21
Platelet count (10^9^/L)	137.4 (92.6–179.3)	142.5 (96.4–185.5)	0.72
Size of lesion (maximum diameter, cm)	3.7 (1.4–4.8)	3.3 (1.7–4.6)	0.31
HCC	72 (65.5)	38 (64.4)	0.89

*Note.* Except where indicated, data are numbers of patients, with percentages in parentheses. ^*a*^Data are medians, with interquartile range in parentheses.

**Table 2:** Diagnostic performances of radiomic signature and index for distinguishing HH and HCC in the training and validation group.

	Training group		Validation group	
	Radiomic signature	Radiomic index	Radiomic signature	Radiomic index
AUROC	0.792	0.88	0.716	0.87
CI	(0.703, 0.882)	(0.817, 0.943)	(0.581, 0.85)	(0.782, 0.957)
Cutoff	−0.267	0.608	0.026	1.942
Sensitivity	0.764	0.806	0.579	0.605
Specificity	0.737	0.816	0.857	1
Positive predictive value	0.846	0.892	0.88	1
Negative predictive value	0.622	0.689	0.529	0.583
Correctly classified	0.755	0.809	0.678	0.746
Comparison of AUROC	*P* = 0.014	*P* = 0.003		

*Note.* AUROC: area under the receiver operating characteristics; CI: confidence interval.

**Table 3:** Multivariate analysis of radiomic features for discriminate HH and HCC.

Variables	*b* coefficient	Hazard ratio	*P* value
Original-shape-volume	NA	NA	0.371
Wavelet-LLL-first-order-median	0.687	1.987 (1.039–3.799)	0.038
Wavelet-LLL-gldm-small-dependence-low-gray-level-emphasis	NA	NA	0.720
Wavelet-LHL-glszm-zone-entropy	−2.165	0.115 (0.042–0.311)	<0.001
Wavelet-LLH-glszm-zone-entropy	NA	NA	0.888

*Note. b* coefficients are from multivariable logistic regression. HH, hepatic hemangioma; HCC, hepatocellular carcinoma.

## Data Availability

The datasets analyzed during the current study are available from the corresponding authors on reasonable request.
